# Ethnic Music Inheritance and Environmental Monitoring Using Big Data Analysis from the Cultural Perspective

This article has been retracted.

**DOI:** 10.1155/2022/2485596

**Published:** 2022-10-08

**Authors:** Jian Cui, Karin Khomkrich

**Affiliations:** College of Music, Mahasarakham University, 44000, Thailand

## Abstract

Ethnic music has too many expectations due to its significance to the national culture. It serves as a mirror, reflecting all the true characteristics of many geographical areas and ethnic groupings. Instilling national self-confidence and fostering national unity are essential outcomes of this. The optimal design plan for Xinjiang folk music inheritance and environmental monitoring based on big data technology is presented in this study from the standpoint of cultural ecology. Big data technology can categorize users who are interested in Xinjiang ethnic music, and after that, through customized recommendation filtering, consumers may be presented with Xinjiang ethnic music that meets their interests. Last but not least, a simulation test and analysis are performed. The algorithm's accuracy is 7.86% higher than that of the conventional algorithm, according to the simulation data. By studying and calculating the user's behavioral traits and interests, this result demonstrates in detail how the recommender system can display the user's content efficiently. However, there are numerous possibilities and varied contexts for the use of clustering techniques in recommender systems. It is crucially vital for directing the protection of ethnic music and fostering the inheritance and development of ethnic culture to conduct design study on the Xinjiang region's ethnic music heritage and development with cultural ecology as the central guiding principle. This article is from “A comprehensive study of Uygur Muqam music art with Chinese characteristics,” which aims to improve the data reserve of the world and Southeast Asia on the research of Chinese Uighur Muqam art. Improve the inheritance and development of music in Xinjiang, China, and provide more detailed data to more scholars. This study adopts qualitative research methods and field survey data. The author proposes to focus on the perspective of cultural ecology, based on the use of big data technology, to improve the inheritance and development of Xinjiang national music.

## 1. Introduction

Xinjiang is located in the northwest border of China. There are 13 ethnic groups living in this land, including Han, Uygur, Kazak, Mongolian, and Xibe. The unique geographical location makes Xinjiang and the East and West have frequent ethnic migration and cultural exchanges since ancient times [1]. Each nation has formed its own cultural symbols in the process of historical integration and cultural differentiation and reorganization and has been handed down from generation to generation [2]. Productive labor is the material basis for human survival and development [3]. With the acceleration of the modernization process, the inherent mode of production and labor on which people live has undergone tremendous changes, leading to fundamental changes in living customs [4]. And the original ecological folk songs are closely related to people's production and life. Those traditional music genres that rely on specific production labor have lost their foundation for continued existence due to the change of production mode. With the accelerated development of China's economy, the replacement of agricultural civilization by industrial civilization has led to the destruction of agricultural culture. The natural environment and social environment that originally adapted to agricultural culture have also undergone dramatic changes, resulting in a great threat to the survival of the national traditional culture, especially the minority music culture. With the development of the western region and the economy, great changes have taken place in Xinjiang's traditional music culture. Many music forms are disappearing because they cannot adapt to the changes of the environment. Therefore, how to protect, spread, and develop Xinjiang national folk music culture in the perspective of cultural ecology has become an urgent issue [5].

Cultural ecology is a science that studies the relationship between culture and environment. It is an interdisciplinary subject of culturology and ecology. It studies the process of a society adapting to its environment. Its main problem is to determine whether these adaptations cause internal social changes or progressive changes. The theory of cultural ecology generally believes that culture is not directly influenced by a certain factor, but appears under the cross influence of multiple complex variables [6]. Culture is the result of how man and nature work together, according to cultural ecology. A certain national, regional, historical, and other characteristics must be present in the culture that emerged during a particular historical time. It is a cultural mode and state with ecological flexibility, reciprocal influence, and mutual restriction of different factors in a certain historical time. The amount of data generated by people's production activities will increase as Internet technology continues to advance, and data and people's daily lives will become more and more intertwined. People can discover other hidden rules from these vast amounts of data through analysis and processing, which will aid in the evolution of the entire society. Big data application technologies [7, 8], such as different big data platforms, big data index systems, and other big data application technologies, are referred to as big data technology. On the one hand, big data technology is connected to a variety of industries, and its application promotes the general advancement of society. On the other hand, in order to facilitate decision-making, the development demands of every sector of society also require the acquisition of additional data by technical methods, as well as data mining and analysis. Big data technology is created and developed as a result of social development demands. In light of the benefits of big data technology, this study applies the filtering method to lower the cost of arithmetic execution. It has been demonstrated via practice that this combination can enhance the quality and effectiveness of Xinjiang ethnic music inheritance and development optimization in addition to shortening calculation times.

Cultural ecology emphasizes analyzing the relationship between culture and environment from the perspective of culture and region [9]. There is also a complex relationship between these factors [10]. In traditional music, different cultural states have different positions and functions, which jointly build the cultural foundation of Xinjiang ethnic music and form the cultural uniqueness under specific natural environment and regional characteristics [11]. Xinjiang is a region rich in resources. In the course of development for thousands of years, ethnic music reflects the characteristics of people's lives. Although the languages of different ethnic groups are different, and each ethnic group has its own tonal system, its musical creativity and penetration are very significant, with a unique cultural background. The openness of the state in ethnic and religious policies also provides spiritual support for the inheritance of ethnic music. Since ancient times, such music development trend conforms to the law of social and historical development, and national music can also reflect its important artistic characteristics.

In this paper, a feature reconstruction model of Xinjiang ethnic music inheritance and development optimization design is established. Aiming at the problem of data sparsity in collaborative filtering arithmetic, by analyzing user interest points, clustering arithmetic is applied to user based music collaborative filtering recommendation to cluster users. Its innovation lies in the following:

1. This paper adopts the filtering method in big data technology to reduce the execution cost of the arithmetic
2. This paper constructs the key feature quantity of Xinjiang ethnic music inheritance and development optimization design and adopts personalized recommendation technology to realize the optimization design and identification of Xinjiang ethnic music inheritance and development

## 2. Related Work

It is found in the current research and literature collation that Xinjiang ethnic music is actually a potential innovative form that integrates and infiltrates with other relevant specific contents of the cultural industry, realizing its cultural meaning and economic value as a support for national cultural identity, national cultural industry development, etc. [12].

Zhang et al. discussed the countermeasures for the continuous inheritance of modern school music education from different angles, the importance of national folk music in the world music culture, and pointed out that music is an important content in the national cultural inheritance, and national music is an important factor related to national consciousness and national prosperity [13]. Mellor et al. put forward in the preservation and development of the traditional music of all ethnic groups in Xinjiang: “to cultivate the successor talents of the traditional music of all ethnic groups, we should adopt the method of combining symbolic recording and oral and mental teaching to ensure the comprehensive inheritance of the traditional music wealth held by teachers, and professional workers should not give too much guidance and intervention” [14]. Lakshmanaprabu and others mentioned “the inheritance of local music culture and the current situation of music education in Xinjiang, the thinking on the current situation of local music education, and the basic ideas and methods of local music curriculum construction.” It can be seen that Xinjiang, a multiethnic region, is rich in music resources. Local music resources are added to school education to enrich the curriculum content of music education [15]. Yan systematically described the source, composition, artistic characteristics, and development of Chinese traditional music and, compared with western music, elaborated the representative music types and tonal characteristics of various systems and branches of Chinese traditional music [16]. Lowerre Barbieri and others have classified and studied Xinjiang's ethnic music from many aspects such as “folk songs,” “folk musical instruments,” “folk instrumental music,” “opera music,” “quyi music,” and “religious music.” On the basis of musicology, they have presented us with a detailed description of Xinjiang's ethnic music [17]. Bestelmeyer and others pointed out that Xinjiang's national music is the spread of spiritual culture, the normative strengthening of institutional culture, the transmission of wisdom of labor culture, the expression of communication culture, and the memory call of historical culture [18]. Callaghan et al. proposed that music is not an isolated social existence. With the changes of social life and the different needs of human self-development, the meaning and mode of music are constantly enriched and updated [19]. Bernetti and others, taking the Xianzu as an example, explored the cultural significance of the original ecological music by using TV and other media means to make it conform to the characteristics of the current consumer society, so as to create its unique cultural advantages through its personalized advantages [20]. Bhatia pointed out the following: In the process of globalization, national culture faces the danger of being converged and homogenized. In order to survive and develop in the constantly changing environment, it is necessary to create opportunities and impetus by virtue of the diversity and heterogeneity of culture itself, consciously self-renew and self-transform the traditional culture of the nation, and continue and evolve [21].

Currently, when Xinjiang ethnic music is discussed, its artistry, culture, and diversity as music have all been completely acknowledged and expounded upon, as well as certain current phenomena. However, other than its fundamental relevance, the evolution of Xinjiang ethnic music has not been specifically integrated and analyzed from the perspective of cultural ecology. From the standpoint of cultural ecology, this research suggests an optimum design strategy for the transmission and evolution of Xinjiang ethnic music based on big data technology. It gathers complete information on user interests using user big data collection techniques, laying the groundwork for tailored recommendation. Utilize clustering to group user data with similar interest patterns, big data analysis to identify user interests, and independent sampling based on big data to enhance model generalization performance and avoid overfitting.

## 3. Methodology

### 3.1. Personalized Analysis of Xinjiang Folk Music Users Is Recommended

Xinjiang ethnic minority region is one of the main areas in which we study music education in ethnic minority regions. Therefore, Xinjiang ethnic minorities have become a development model of multicultural music [22]. The inheritance status of Xinjiang ethnic music in the perspective of cultural ecology is worth investigating and studying. It has fundamentally changed with the traditional folk artists in the way of “oral and heart to heart transmission” [23]. The excellent national cultural heritage was passed on through education, and the inheritance was strengthened. The excellent national culture was carried forward, and the national music education was brought into a standardized and localized music education system.

To ensure that ethnic music from Xinjiang keeps up with the times, we can employ tailored recommendation technologies to understand the demands of users. The ability to offer customized services without knowing the exact needs of the user is the most crucial aspect of a personalized recommendation system. The fundamental idea behind recommendations is to first evaluate previous data to determine the user's interest and then to present the user with recommendations that match that interest. Because of this, the recommendation system helps users find satisfying services and is in demand. In the recommendation system, users interact with the system via the front-end interface, and the system records their operation behavior and other data to create and store a log. The recommendation algorithm analyzes these data to produce recommendation results, which are subsequently displayed to the user on the front-end page.  Figure 1 displays the recommended system's typical architecture.

The Xinjiang ethnic music personalized recommendation system is analyzed in detail, the design objectives are determined, the system requirements are clear, and the design process is completed. Combined with the traditional music recommendation process, the business process of this system is analyzed. The business process of the recommendation process is shown in Figure 2.

The first is data collection. Traditional recommendation systems mainly use log data to obtain user behavior data. The amount of data obtained in this way is small, and the dimension is low. In order to obtain the big data of the recommendation system, this paper adds data sources such as databases, sensors, and network interfaces on this basis. In addition to user behavior data, it also collects original data such as user attribute data, behavior context data, and music work data. The next step is to calculate and generate a recommendation list. Traditional music recommendation systems generate recommendation results by calculating the similarity of user behavior. In the big data environment, this method is not accurate enough to grasp the user's interest, and the data processing ability cannot meet the requirements. In this study, the data are preprocessed to make them available for calculation. Then, the recommendation list is generated by using the music personalized recommendation method introduced in Chapter 3. The calculation of this process adopts MapReduce framework and is implemented in Hadoop cluster. It not only ensures the potential value of user data, but also improves the system's computing capacity. The last step is data embedding. After calculating and obtaining the music personalized recommendation method, save these data in the database, and embed the recommendation results into the web service.

Collaborative filtering, which is based on information on user activity, is the most popular method used in recommendation systems. The basic principle that “birds of a feather flock together and people flock together” lies at the heart of collaborative filtering arithmetic. It is mostly used to determine how similar things and users are. The most traditional and developed recommendation arithmetic is collaborative filtering arithmetic. The scientific research community has developed numerous methodologies as a result of a number of in-depth study findings. Among these, the traditional approaches include the neighborhood approach, the cryptic meaning approach, and the graph-based random walk approach. The most well-known and frequently employed strategy in the sector is the neighborhood-based recommendation method. The two primary categories of neighborhood-based suggestions are as follows:

1. User-based collaborative filtering: user-based CF recommends items similar to user preferences to target users
2. Collaborative filtering based on items: Item-based CF recommends items similar to their favorite items for target users. User-based collaborative filtering user based CF is the oldest arithmetic in the field of recommendation research. The process of collaborative filtering and recommendation based on users is to find other users' favorite items similar to the target users and finally recommend the items that meet the needs of the target users. It mainly includes two steps: finding user sets similar to user interests, count the items that the user likes in the previous step to form a collection, and remove the items that the target user has interacted with, and the rest is the recommendation result

The key of the user based CF arithmetic is to analyze the user behavior and calculate the similarity between the target user and other users, which is usually obtained by behavior similarity calculation. For example, the two users *u* and *v* first define *N*(*u*) to represent the collection of items *u* that have expressed their preferences in the past, and *N*(*v*) to represent the collection of items *v* that have expressed their preferences in the past. The similarity of interests between the users *u*, *v* can be calculated by using *N*(*u*) and *N*(*v*). Researchers have invented many formulas to calculate the similarity of user interests. For example, Formula (1) can roughly obtain the similarity of interests between the user *u* and the user *v*:

(1) $$\begin{array}{c} w_{uv}=\frac{\left|N\left(u\right)\cap N\left(v\right)\right|}{\left|N\left(u\right)\cup N\left(v\right)\right|}. \end{array}$$

The cosine similarity Formula (2) can also be used for calculation:

(2) $$\begin{array}{c} w_{uv}=\frac{\left|N\left(u\right)\cap N\left(v\right)\right|}{\sqrt{\left|N\left(u\right)N\left(v\right)\right|}}. \end{array}$$

The similarity calculation between any users can be completed by the above formula. The time complexity of the two methods is as high as *O*(*N*^2^) in theory. However, in fact, for one kind of music, the behavior will not occur in all users, and |*N*(*u*)∩*N*(*v*)| is usually 0.

### 3.2. Optimization of Xinjiang Ethnic Music Recommendation Based on Big Data Technology

The survival and growth of national music against the backdrop of multicultural is experiencing significant challenges in the era of global economic integration. The rise of mass media has also altered how individuals consume culture and what they need spiritually. But we must learn from difficulties and accurately comprehend how national music and contemporary culture are related. Blindly emphasizing the originality of ethnic music is not in accordance with the rule of social evolution. Due to its natural hereditary features, ethnic music is neglected and continues to exist in this way.

For processing massive amounts of data, Hadoop is an open source computing system based on Java. Hadoop has two primary structural components as a distributed big data processing platform. One of them is Hadoop Distributed File System (HDFS), which enables centralized file management across distributed computers. Additionally, HDFS uses a distributed file system with a master-slave hierarchy. Hadoop cluster consists of several slave nodes and a master node. Another component is the MapReduce calculation engine, which facilitates distributed data calculation. To do this, a work is first broken up into numerous smaller tasks, and then the results are combined as necessary to speed up data processing. When a client needs to write, the namenode receives the file write request and checks the datanode information it manages on its own to see if it is appropriate for writing. If it is appropriate for writing, it will send the client writable data in accordance with its configuration and the size of the file that needs to be written, after which it will allow the client to perform the file blocking operation and write in accordance with the address information provided by the datanode. When the client has to read, it is simpler. In a similar manner, the client must first send a read request to the namenode. The namenode can directly return the information stored in the datanode for the client to read the file.

The point of interest data is used to analyze the degree of aggregation and mixing of various functional formats. The former was analyzed by nuclear density and the latter by point statistics.

#### 3.2.1. Nuclear Density Analysis

Nuclear density analysis can be used to examine the spatial properties of point data distribution, investigate concentrated areas of sample distribution, and visually represent the degree and distribution of different functional formats.

#### 3.2.2. Point Statistical Analysis

Point statistical analysis can calculate the average value, maximum value, minimum value, standard deviation, total value, type, etc. of each pixel of grid data within a certain range and can calculate the types of business forms included within a certain range, that is, their diversity, and visualize them. To import the data of interest points into ArcGIS software, firstly, the coordinate converter is used to change the data of interest points into spatial data using longitude and latitude coordinates; And then display the data in the form of dots according to the longitude and latitude information; Finally, we use nuclear density analysis tools to analyze the degree of aggregation of different types of business forms and point statistical analysis tools to analyze the degree of functional mixing in a certain area, wherein the kernel density function is

(3) $$\begin{array}{c} \hat{f}\left(x,y\right)=\frac{3}{{nh}^{2}\pi }\overset{n}{\underset{i=1}{\sum }}w_{i}{\left\{1-{\left(\frac{\sqrt{{\left(x-x_{i}\right)}^{2}+{\left(y-y_{i}\right)}^{2}}}{h}\right)}^{2}\right\}}^{2}, \end{array}$$

where $\hat{f}\left(x,y\right)$ represents the kernel density of data, (*x*_*i*_, *y*_*i*_) represents *n* sample points distributed independently, and *h* is the smoothing parameter.

This method is used to calculate the music interest preference and kernel density of the POI data as quantitative indicators of the degree of functional mixing and the degree of functional aggregation.

## 4. Result Analysis and Discussion

Music is an important part of culture. Its development is closely related to the natural environment and social environment. Thanks to the rich natural resources, the creation and development of Xinjiang ethnic music has very rich resources and inspiration. Nurtured by the unique ecological environment in Xinjiang ethnic areas, Xinjiang ethnic original ecological music can be preserved and continued. On the one hand, since the reform and opening up, foreign music culture has been introduced one after another. Traditional Xinjiang national music is impacted by foreign music. More and more young people turn to western music for learning and research. The inheritors of national music are aging gradually, and Xinjiang national music is also facing the crisis of losing. On the other hand, many ethnic minority areas in Xinjiang have relatively difficult living conditions, inconvenient road traffic, fewer ethnic groups, backward economic conditions, and relatively closed environment. This gap between economic and environmental conditions also makes the development of music culture of these nationalities more difficult. This is an urgent problem to be studied and solved in the inheritance and development of Xinjiang ethnic music culture.

Test the proposed method's processing time requirements with various users. Assign separate user numbers to this method's and the other two's execution times. By comparing the execution times, the method's processing efficiency is confirmed. The experimental data came from the millions of songs dataset. This data has a wide range of dimensions, making it particularly useful for confirming tailored music recommendation algorithms. Additionally, it offers a sub-dataset that includes information about users and music works as well as activity data records for roughly 20,000 people across 100,000 pieces of ethnic music from Xinjiang.

K- means clustering arithmetic is a very widely used clustering arithmetic in the field of big data. Because of its computational process characteristics, it has strong independence and can be distributed to different nodes, without the need for each node to cooperate. Therefore, the *K* value is introduced into the arithmetic in this paper, because the selection of *K* value will also affect the classification results and ultimately affect the effect of the recommended arithmetic. After repeated experiments, the changes of accuracy and recall on *K* value are shown in Figure 3

According to Figure 3, which compares the accuracy of the two arithmetics' suggested results, the K-means clustering arithmetic is more accurate than the conventional collaborative filtering arithmetic based on users. The accuracy increases by around 0.79 percent when the *K* value is 8, producing the greatest results at this time. The recommendation impact after K-means clustering is introduced is generally superior to the conventional collaborative filtering recommendation arithmetic based on users.

Figure 4 is a change diagram of the recall rate of the two arithmetics. After introducing the K-means clustering arithmetic, the accuracy rate is better than the traditional collaborative filtering arithmetic based on users. When the *K* value is 8, the recall rate can be improved by about 0.81%. Because when the number of users is fixed, after removing the free points, each classification will be affected, and the number of some classifications is very small, so the recommendation result is not accurate, thus affecting the overall recommendation arithmetic effect. It is similar to Figure 4, because the number of recommended songs for each user is similar to the number of songs in the user's test set when the number of recommended songs is given to the user, so the trend of recall and accuracy is also similar.

The results of the experiment will be discussed and provided in this article. The processing effectiveness of the approach is initially evaluated. The user-based and item-based methods to CF are contrasted with the suggested recommended approach. The figure comparing processing times is shown in Figure 5 below. When there are less than 180 users, the personalized recommendation approach proposed in this research performs slower than the traditional user-based CF and item-based CF methods. This is because the Hadoop platform requires some setup and startup time and there is also visible cost from distributed computing. Until the user scale is greater than 160; however, the execution speed is faster than the traditional user-based CF and item-based CF techniques. With more data being generated, the research's proposed technique also offers more obvious computational benefits.

A comparison of the three approaches' suggested results' accuracy is shown in Figure 6. The findings shown in Figure 6 demonstrate that the recommendation approach suggested in this research has a clear advantage when comparing the precision of the suggestion outcomes. The accuracy rate is roughly 7% greater than that of the conventional method after the user data reaches a specific level. The performance of this method is superior than the conventional method regardless of the user count since it pulls on and integrates the recommendation concepts of the two fundamental methods. Furthermore, as the user base grew, the accuracy of the suggestion results steadily stabilized and finally rose to above 30%.

The three techniques' coverage of the suggested results is shown in Figure 7. The coverage rates of the three techniques steadily decline as the total number of users rises, according to the information in the graph. In any event, the proposed approach is much more coverage-efficient than the conventional user-based CF and item-based CF approaches tested in this study.

In summary, the processing performance, accuracy rate, and coverage rate of the suggested technique in this study are superior to those of the conventional method. In any event, it is better than the conventional approach. It demonstrates how this way of recommending musical works might anticipate a user's preferences and reduce frequent problems with the recommendation system when compiling the user's final suggestion list.

## 5. Conclusion

From the standpoint of cultural ecology, this research suggests an optimum design strategy for the transmission and evolution of Xinjiang ethnic music based on big data technology. Via the use of big data technology, it categorizes interested listeners of Xinjiang ethnic music, and through the use of personalized suggestion filtering, it then offers consumers Xinjiang ethnic music that suits their interests. The simulation test and analysis are done in the end. According to the simulation findings, the proposed arithmetic has an accuracy that is 7.86% higher than that of the conventional arithmetic. This outcome demonstrates in full how the recommendation system, by evaluating and calculating the user's behavior features and interests, may display the user's content in an effective manner. In addition, there are many different applications for clustering mathematics in the recommendation system. The national music culture of Xinjiang is a priceless relic from the long river of national history. We must improve the management and preservation of Xinjiang's national ecological environment, raise the awareness of people from all nationalities to preserve Xinjiang's national music, delve deeply into the stirring voices left in the mountains, assist Xinjiang's national music in gradually moving to the forefront of the cultural industry development stage, and encourage more people to appreciate Xinjiang's national music. In the process of adapting to the cultural and social environment, the traditional elements are also continuously inherited and innovated. How to adapt to the cultural ecological law is also the main direction of the future development of national music. In the future research work, we should further analyze the cultural composition of music elements from the perspective of cultural ecology and combine the main characteristics of the development of Xinjiang ethnic music to achieve culture and inheritance and development.

## Figures and Tables

**Figure 1:** Common architecture of recommendation system.

**Figure 2:** Business flow chart of recommendation process.

**Figure 3:** Change of accuracy of the two arithmetics with the number of classification *K*.

**Figure 4:** Change of the recall rate of the two arithmetics with the number of classification K.

**Figure 5:** Comparison of execution time of recommended methods.

**Figure 6:** Comparison of accuracy of recommendation results.

**Figure 7:** Comparison of recommended results coverage.

## Data Availability

The data used to support the findings of this study are available from the corresponding author upon request.

## References

[1] Ma A., Bohan D., Canard E. (2018). A replicated network approach to ‘big data’ in ecology. *Advances in Ecological Research*.

[2] Whitaker A. R., Rosenthal J. S., Brandy P. (2019). Social boundaries, territoriality, and the cultural ecology of artiodactyl hunting in prehistoric Central California. *Quaternary International*.

[3] Zhao M., Zhao S. C., Zhang L. Y. (2017). Applications of eco-environmental big data: progress and prospect. *Journal of Applied Ecology*.

[4] Joseph M., Stone M. A., John K. (2018). Application of data mining to a large hearing-aid manufacturer’s dataset to identify possible benefits for clinicians, manufacturers, and users. *Trends in hearing*.

[5] David G., Damien C., Christophe G. (2022). Big data approaches to the spatial ecology and conservation of marine megafauna. *ICES Journal of Marine Science*.

[6] Benedetti-Cecchi L., Bulleri F., Bello M. D. (2018). Hybrid datasets: integrating observations with experiments in the era of macroecology and big data. *Ecology*.

[7] Pan H., Zheng L. (2022). N-SVRG: stochastic variance reduction gradient with noise reduction ability for small batch samples. *CMES-Computer Modeling in Engineering & Sciences*.

[8] You L., Jiang H., Hu J. GPU-Accelerated Faster Mean Shift with Euclidean Distance Metrics.

[9] Li L., Liu X., Du R. (2018). Application of big data technology in evaluation of operating status of high-pressure hydrogenation heat exchanger. *China Petroleum Processing and Petrochemical Technology*.

[10] Xu D. (2020). Research on music culture personalized recommendation based on factor decomposition machine. *Personal and Ubiquitous Computing*.

[11] Ranga K. K., Nagpal C. K. (2022). A big data analytics framework for determining the travel destination preferences of Indian tourists. *International Journal of Modern Physics C*.

[12] Ergashev I., Farxodjonova N. (2020). Integration of national culture in the process of globalization. *Journal of Critical Reviews*.

[13] Zhang H., Guo T., Su X. (2021). Application of big data technology in the Impact of tourism E-commerce on tourism planning. *Complexity*.

[14] Mellor J. C., Stone M. A., John K. (2018). Application of data mining to "big data" acquired in audiology: principles and potential. *Trends in Hearing*.

[15] Lakshmanaprabu S. K., Shankar K., Rani S. S. (2019). An effect of big data technology with ant colony optimization based routing in vehicular ad hoc networks: towards smart cities. *Journal of Cleaner Production*.

[16] Yan S. (2020). The perception difference analysis of the influence of coastal residents of big data mining technology on marine tourism development. *Journal of Coastal Research*.

[17] Lowerre-Barbieri S. K., Catalan I. A., Opdal A. F. (2019). Preparing for the future: integrating spatial ecology into ecosystem-based management. *ICES Journal of Marine Science*.

[18] Bestelmeyer B. T., Spiegal S., Winkler R., James D., Levi M., Williamson J. (2021). Assessing sustainability goals using big data: collaborative adaptive management in the Malpai Borderlands. *Rangeland Ecology & Management*.

[19] Callaghan C. T., Sayol F., Benedetti Y., Morelli F., Sol D. (2021). Validation of a globally-applicable method to measure urban tolerance of birds using citizen science data. *Ecological Indicators*.

[20] Bernetti I., Chirici G., Sacchelli S. (2019). Big data and evaluation of cultural ecosystem services: an analysis based on geotagged photographs from social media in Tuscan forest (Italy). *Forest-Biogeosciences and Forestry*.

[21] Bhatia S., Priya K. R. (2018). Decolonizing culture: Euro-American psychology and the shaping of neoliberal selves in India. *Theory & Psychology*.

[22] Bai X., Li J. (2021). Personalized dynamic evaluation technology of online education quality management based on artificial intelligence big data. *Journal of Intelligent and Fuzzy Systems*.

[23] Wu J., Wang J., Nicholas S., Maitland E., Fan Q. (2020). Application of big data technology for COVID-19 prevention and control in China: lessons and recommendations. *Journal of Medical Internet Research*.

